The article "ECG Signal Modeling Using Volatility Properties: Its Application in Sleep Apnea Syndrome" was published in 2021. Journal: J Healthc Eng.

# ECG Signal Modeling Using Volatility Properties: Its Application in Sleep Apnea Syndrome

**DOI:** 10.1155/2021/4894501

**Published:** 2021-07-07

**Authors:** Maryam Faal, Farshad Almasganj

**Affiliations:** Department of Biomedical Engineering, Amirkabir University of Technology, Tehran, Iran

## Abstract

This study presents and evaluates the mathematical model to estimate the mean and variance of single-lead ECG signals in sleep apnea syndrome. Our objective is to use the volatility property of the ECG signal for modeling. ECG signal is a stochastic signal whose mean and variance are time-varying. So, we propose to decompose this nonstationarity into two additive components; a homoscedastic Autoregressive Integrated Moving Average (ARIMA) and a heteroscedastic time series in terms of Exponential Generalized Autoregressive Conditional Heteroskedasticity (EGARCH), where the former captures the linearity property and the latter the nonlinear characteristics of the ECG signal. First, ECG signals are segmented into one-minute segments. The heteroskedasticity property is then examined through various tests such as the ARCH/GARCH test, kurtosis, skewness, and histograms. Next, the ARIMA model is applied to signals as a linear model and EGARCH as a nonlinear model. The appropriate orders of models are estimated by using the Bayesian Information Criterion (BIC). We assess the effectiveness of our model in terms of mean square error (MSE), root mean square error (RMSE), mean absolute error (MAE), and mean absolute percentage error (MAPE). The data in this article is obtained from the Physionet Apnea-ECG database. Results show that the ARIMA-EGARCH model performs better than other models for modeling both apneic and normal ECG signals in sleep apnea syndrome.

## 1. Introduction

ECG signal has an essential role in medical diagnosis for the study of cardiac function and abnormalities. Considering the abnormal activity of heart or heart rate variation (HRV) could be an indicator of some diseases such as congestive heart failure (CHF) [1], sudden cardiac death (SCD) [2], and obstructive sleep apnea (OSA) [3]. OSA is a common respiratory disease characterized by a cessation in the airflow for at least 10 seconds [4]. The literature has stated that sleep apnea affects approximately 2% of women and 4% of men and that most of them are overweight [5]. Apnea increases accidents and mortality rates. Previous research considered apnea as a public health risk compared with smoking. Untreated OSA can also cause depression, high blood pressure, stroke, hypertension, death, and an increased risk of long-term and short-term disease. It increases the risk of myocardial infarction by up to 20% and heart attack by up to 40% [6]. Accurate and early diagnosis is an essential step in the control and prevention of sleep apnea. So, it attracts much attention in ECG research.

The article "ECG Signal Modeling Using Volatility Properties: Its Application in Sleep Apnea Syndrome" was published in 2021. Journal: J Healthc Eng.

Polysomnography (PSG), a multimodality system, is the most accurate and precise method of sleep monitoring, which can be used to describe sleep stages and disorders. PSG measures electrocardiogram (ECG), electroencephalogram (EEG), electromyogram (EMG), electrooculogram (EOG), and respiratory airflow and peripheral oxygen saturation (SpO2). After collecting the PSG data, physicians rate the OSA events using statistical methods. The PSG system, on the other hand, has two major defects. First, manually scoring sleep stages according to the guideline requires the use of physicians and appropriate sensors is time-consuming and expensive. Therefore, PSG can only be performed in sleep laboratories, which delays detection and results in a long waiting list. Second, it is an obtrusive approach, which requires the attachment of several sensors and wires. Sleep normality can be disrupted by the sensors and wires, making PSG inappropriate for long-term sleep researches [7]. So, developing methods that can accurately detect apnea with a few signals at home is critical. These approaches were focused on biosignals such as respiratory, snoring, SpO2, and ECG signals, and several authors have achieved a high level of performance in terms of OSA detection [8–11].

Using wearable devices with some necessary biosensors for sleep disorder diagnosis is safer because these devices are designed with unobtrusiveness insight. Furthermore, they are simpler to use, easier to find, and less expensive than clinical measurements. The ECG is one of the most reliable physiological signals given by various wearable devices and used in many OSA studies [12]. Several researchers have suggested innovative methods for evaluating sleep quality and sleep apnea using only a single-lead ECG. The presence of irregular characteristics in the ECG signal is seen as a warning sign of sleep apnea. When sleep apnea occurs, the oxygen saturation decreases and the cardiovascular system is activated to maintain the oxygen intake constant. Furthermore, according to a clinical study in [7], patients' compliance is extremely low when wearing the pressure transducer sensor to achieve nasal and oral respiration. Patients usually pulled out the nasal cannula and nasal airflow data can be unreliable compared to the ECG signal due to lead loss. As a consequence, we chose ECG signals to model OSA and normal events in this study.

The majority of ECG approaches proposed in the literature for sleep apnea detection are based on feature extraction from single-lead ECG signals and using classifiers [8–11]. Zarei and Mohammadzadeh Asl [10] proposed a novel approach based on single-lead ECG autoregressive (AR) modeling and ECG feature extraction using the spectral autocorrelation function. Sequential forward feature selection (SFFS) is used to select the most appropriate features, which are then fed into a random forest to classify normal and apnea epochs. Singh et al. [8] extracted the mean and the standard deviation from the instantaneous amplitude (IA) and instantaneous frequency (IF) of each reconstructed component (RC) of heartbeat intervals and electrocardiogram-derived respiration (EDR) signals. Then, stacked autoencoder-based deep neural network (SAE-DNN) and support vector machine (SVM) are used to categorize apneic and normal segments. Zhang et al. [11] suggested a sleep monitoring model based on a single-channel electrocardiogram using a convolutional neural network (CNN). Rajesh et al. [9] extracted moments of power spectrum density, waveform complexity measures, and higher-order moments from the 1 min segmented ECG subbands obtained from discrete wavelet transform (DWT). The acquired feature set is fed to various classifiers such as SVM, linear discriminant analysis (LDA), random forest, and *k* nearest neighbors (kNN). All of these methods are purely data-driven.

The article "ECG Signal Modeling Using Volatility Properties: Its Application in Sleep Apnea Syndrome" was published in 2021. Journal: J Healthc Eng.

Signal modeling and feature extraction is an essential step in the analysis of the ECG signals. Mathematical modeling of the ECG signal is widely used in many cardiovascular studies, such as ECG signals denoising, ECG beats segmentation, arrhythmias detection, heart rate estimation, and synthetic ECG signal generation [13, 14]. Mathematically, modeling helps to understand how the model's factors influence the sensitivity and specificity in computer-aided diagnosis methods. Different models have been used for ECG signals such as autoregressive (AR) model [15], autoregressive moving average (ARMA) [16], generalized autoregressive moving average (GARMA) [17], data flow graph (DFG) model [18], generalized orthogonal forward regression (GOFR) [19], Gaussian mesa and bi-Gaussian functions [19], hidden Markov models (HMM) [20], morphological models [21], Hermite basis functions [22], Gaussian model [23], principal component analysis [24], Kalman filter [25], and time-varying autoregressive model (TVAM) [26]. These ECG models have fitted mathematical representations into HRV or the points of ECG signals and need ECG preprocessing to achieve essential components such as QRS complexes, P-wave, and T-wave. The main drawback is that using these components needs to determine the exact location of waves, which increases the computation time, and the system performance depends on the method used. Therefore, in this article, we used an unprocessed single-lead ECG signal, which is lower in cost. Only a few researchers used models to detect apnea [26–28]. Mendez et al. [26] used a time-varying autoregressive model (TVAM) to assess power spectral densities for the QRS complex area and the RR intervals. This study aims to use time series models to propose a new ECG signal model. This model can be used to detect normal and apneic ECG signals. Sharma and Sharma [27] used a linear combination of the lower order Hermite basis functions to estimate each QRS complex of the ECG signal. Hassan et al. [28] used a tunable-Q factor wavelet transformation (TQWT), and each subband was modeled using symmetric Normal Inverse Gaussian (NIG) pdf. One issue neglected in previous articles is that apnea is associated with fluctuations in the ECG process. This property can be used to model apnea and normal ECG signals.

The article "ECG Signal Modeling Using Volatility Properties: Its Application in Sleep Apnea Syndrome" was published in 2021. Journal: J Healthc Eng.

Time-varying conditional standard deviation, usually called volatility, describes periods of high oscillations distributed with relative calm periods and plays a vital role in predicting time series fluctuations [29]. In statistics, heteroskedasticity indicates that a variable standard error is not constant over time. It has been proven that heteroskedasticity modeling through Autoregressive Conditional Heteroskedasticity (ARCH) and Generalized Autoregressive Conditional Heteroskedasticity (GARCH) and their variants are helpful in the modeling varying volatility in nonstationary time series [29]. Real-world time series such as ECG signals have volatility. In the literature, ECG volatility and heteroskedasticity during apnea are underestimated. Huand Tsoukalas [30] showed that Integrated GARCH(1, 1) could model apneic ECG segments, and ARCH(1) can model the normal ECG recordings. Experimental observations showed that cardiovascular variations are complex, nonlinear, and nonstationary [31]. Linear models like AR, Moving Average (MA), and ARMA are coarse estimations of real-world systems and usually have poor performance in forecasting the evolution of nonstationary and nonlinear processes [31]. The ARIMA model is usually used to model these patterns [31]. Therefore, in this article, the ARIMA model is used to model linear features of ECG signals. The consistency of conditional variance is one of the essential assumptions used by conventional ARIMA models to forecast future values. If we assume that the ARIMA model fits an ECG signal, the conditional variance should be constant. It has been shown that during apnea, the homoskedasticity assumption is not correct [29]. Instead of using the ARIMA model, which focuses only on predicting the conditional mean of future values, clusters of abundant variance need to use models that can simultaneously predict both the conditional mean and the conditional heteroscedasticity of the system. Since ARIMA is a linear model, it cannot reflect nonlinear characteristics such as volatility. ARIMA is a linear model that reveals linear characteristics of the ECG signal, and nonlinear features such as heteroskedasticity of the ECG signal remain in residuals, which are modeled using a nonlinear ARCH or GARCH model. Therefore, the proposed model is based on the linear ARIMA model and a nonlinear GARCH model. First, the heteroskedasticity property of the ECG signal is examined through the ARCH/GARCH test, kurtosis, skewness, and histograms. Next, the linear characteristics of ECG signals are modeled using the ARIMA model. To model the nonlinear heteroskedasticity features of ECG signals, we use three different versions of the original GARCH model: GARCH, Glosten-Jagannathan-Runkle GARCH (GJR-GARCH), and Exponential GARCH (EGARCH). Finally, the model with the maximum likelihood value is selected as the best model among existing models. The best orders of the models are then selected using Bayesian Information Criteria (BIC) and the performance of the proposed model is assessed in terms of four criteria: mean square error (MSE), root mean square error (RMSE), mean absolute error (MAE), and mean absolute percentage error (MAPE).

The article "ECG Signal Modeling Using Volatility Properties: Its Application in Sleep Apnea Syndrome" was published in 2021. Journal: J Healthc Eng.

The article is organized as follows: Section 2 briefly addresses the fundamentals of ARIMA and GARCH models.  Section 3 provides descriptions of the proposed ECG signal model, where data statistic measures and performance metrics are also provided. Associated numerical results are given in Section 4.  Section 5 discusses the obtained results, and the article is concluded in this section, too.

## 2. Prediction Model

In this section, a brief review of the ARIMA and GARCH family models will be presented, respectively.

### 2.1. Autoregressive Integrated Moving Average (ARIMA)

Autoregressive Integrated Moving Average (ARIMA) model is generalized as an ARMA model used in cases where the signal is nonstationary. The ARIMA(*p*, *d*, *q*) model consists of three parts: Autoregressive (AR), Integrated (I), and Moving Average (MA). For a given time series, an ARMA(*p*, *q*) model with *p* as the number of autoregressive terms and *q* as the sum of lagged forecast errors of the following type:

(1) $$\begin{array}{c} \left(1-\sum_{k=1}^{p}a_{k}\right)X_{t}=\left(1+\sum_{k=1}^{q}b_{k}\right)\varepsilon_{t}, \end{array}$$

where *p* is the number of autoregressive (AR) terms, *a*_*k*_*s* are AR parameters, *q* is the number of terms in moving average (MA), *b*_*k*_*s* are MA parameters, and *ϵ*_*t*_ is an independent error term. ARMA models assume that signals are stationary, and the performance of the ARMA model reduces whenever time trends and seasonality features exist. Methods such as ARIMA are used to remove or reduce these nonstationarity moments [32].

The article "ECG Signal Modeling Using Volatility Properties: Its Application in Sleep Apnea Syndrome" was published in 2021. Journal: J Healthc Eng.

The ARIMA model of orders (*p*, *d*, *q*) is a process, *X*_*t*_, whose differences (1 − *L*)^*d*^*X*_*t*_ satisfy an ARMA(*p*, *q*) model, which is stationary. *d* is a nonnegative integer (usually less than (2)) and represents *d*^*th*^ difference of *X*_*t*_ to find a stationary time series. ARIMA models are always assuming the data variance is constant. The following equation can be used to describe the ARIMA(*p*, *d*, *q*) model.

(2) $$\begin{array}{c} \left(1-\sum_{k=1}^{p}a_{k}L^{k}\right){\left(l-L\right)}^{d}X_{t}=\left(1+\sum_{k=1}^{q}b_{k}L^{k}\right)\varepsilon_{t}, \end{array}$$

where *L*{*X*_*t*_}=*X*_*t*_ − *X*_*t*−1_ and *d* is the number of differences required to stationary time series, *a*_*k*_*s* are AR parameters, *p* is the model's autoregression order (AR) and the number of differential series lags, *b*_*k*_*s* are MA parameters, *q* is the order of the model's moving average (MA) and the number of prediction error lags, and *ϵ*_*t*_ is independent error terms. Modeling the ECG signal via ARIMA is essentially a three-stage iterative process that involves the following: identifying model order, model estimation, and checking the model.

### 2.2. Autoregressive Conditional Heteroskedasticity (ARCH) Model

Conditional volatility models are known as heteroscedastic models, meaning the variance is not constant. These models were widely used in finance because data appear to differ or be highly volatile in these areas. Volatility models were first introduced with the Autoregressive Conditional Heteroskedasticity (ARCH) model in economics by Engle [33]. In this model, the conditional variance varies during time as a function of previous errors. Suppose that *Z*(*t*) is a strong white noise process, *Z*(*t*) ~ *N*(0,1); the process *y*_*t*_ can be an ARCH process, if a process is stationary and has the following properties:

(3) $$\begin{array}{c} y_{t}=\sigma_{t}Z_{t},\\ \sigma_{t}^{2}=\alpha_{0}+\sum_{i=1}^{q}\alpha_{i}y_{t-i}^{2}, \end{array}$$

where *Z*(*t*) is a stochastic piece, *σ*_*t*_ is a standard deviation depending on time, *q* is the length of ARCH lags, *α*_0_ ≥ 0, and *α*_*i*_ ≥ 0, * i*=1,2,…, *q*.

### 2.3. Generalized Autoregressive Conditional Heteroskedasticity (GARCH) Model

Although the ARCH method has proven useful in modeling data instability, a relatively long lag is often needed. A simplified version of the ARCH model, i.e., Generalized Autoregressive Conditional Heteroskedasticity (GARCH), was proposed by Bollerslev [34] to allow both longer memory and a more stable lag structure. GARCH modeling is a statistical method for time series modeling whose variances are a stochastic process widely used in modeling financial time series. The main idea of this model is that the conditional variance *σ*_*t*_^2^ has an AR structure and also depends on past values of *σ*_*t*_. GARCH(*p*, *q*) is defined as follows:

(4) $$\begin{array}{c} y_{t}=\sigma_{t}Z_{t},\\ \sigma_{t}^{2}=\alpha_{0}+\sum_{i=1}^{q}\alpha_{i}y_{t-i}^{2}+\sum_{j=1}^{p}\beta_{j}\sigma_{t-j}^{2}, \end{array}$$

where *p* is the order of GARCH terms, *q* is the order of ARCH terms, *α*_0_ > 0, *α*_*i*_ ≥ 0, *β*_*j*_ ≥ 0. The GARCH model's application in various fields proves its ability to model data's uncertainty.

The article "ECG Signal Modeling Using Volatility Properties: Its Application in Sleep Apnea Syndrome" was published in 2021. Journal: J Healthc Eng.

### 2.4. Glosten-Jagannathan-Runkle GARCH (GJR-GARCH) Model

Some more complex GARCH parameterizations were suggested for modeling the conditional variance after the standardized GARCH model. These sophisticated models aim to capture better the empirically demonstrated stylized facts of the mechanism of conditional variance. The asymmetric effect of the negative return shocks, for example, is identified by the Exponential GARCH (EGARCH) model [35] and the Glosten-Jagannathan-Runkle GARCH (GJR-GARCH) model [36]. To conclude, there is no consensus on which GARCH model offers the best for forecasting. Different studies prefer different GARCH parameters, with different study times, different asset groups, and different output assessment requirements. The asymmetric GARCH models are, however, usually favored over the symmetric GARCH model. The first model we used is Glosten-Jagannathan-Runkle GARCH (GJR-GARCH). GJR-GARCH is a nonlinear GARCH model that considers the asymmetries in response to the conditional variance in an innovation. The GJR-GARCH model's principle is that conditional variance dynamics admit that a regime switch depends on the sign of past innovations. It models the asymmetry in GARCH and defined by the following equations:

(5) $$\begin{array}{c} y_{t}=\sigma_{t}Z_{t},\\ \sigma_{t}^{2}=\alpha_{0}+\sum_{i=1}^{q}\alpha_{i}y_{t-i}^{2}+\sum_{j=1}^{p}\beta_{j}\sigma_{t-j}^{2}+\sum_{i=1}^{q}\gamma_{i}I_{t-i}y_{t-i}^{2}, \end{array}$$

where *Z*_*t*_ is i.i.d., *I*_*t*−*i*_=0 if *y*_*t*−*i*_ ≥ 0, and *I*_*t*−*i*_=1 if *y*_*t*−*i*_ < 0

### 2.5. Exponential GARCH (EGARCH) Model

Nelson introduced the Exponential GARCH (EGARCH) (*p*, *q*) model [35] to catch the asymmetry:

(6) $$\begin{array}{c} y_{t}=\sigma_{t}Z_{t},\\ \log\left(\sigma_{t}^{2}\right)=\alpha_{0}+\sum_{k=1}^{q}\beta_{k}g\left(Z_{t-k}\right)+\sum_{k=1}^{p}\alpha_{k}\log\left(\sigma_{t-k}^{2}\right),\\ g\left(Z_{t}\right)=\theta Z_{t}+\lambda \left[\left|Z_{t}\right|-E\left(\left|Z_{t}\right|\right)\right],\\ Z_{t}=\frac{y_{t}}{\sigma_{t}}, \end{array}$$

where *σ*_*t*_^2^ is a conditional variance; *α*_0_, *α*, *β*, *θ*, and *λ* are coefficients. *Z*_*t*_ can be a regular normal variable, or it can come from a generalized distribution of errors. The structure of *g*(*Z*_*t*_) allows for the sign and magnitude of *Z*_*t*_ to have different impacts on the volatility. Since log(*σ*_*t*_^2^) can be negative, the parameters are not subject to sign restrictions.

The article "ECG Signal Modeling Using Volatility Properties: Its Application in Sleep Apnea Syndrome" was published in 2021. Journal: J Healthc Eng.

## 3. ECG Signal Modeling Using ARIMA-EGARCH

ECG signals are segmented into one-minute segments. Each segment has 6000 samples, which contain either normal or apneic conditions. We calculated the order of the models from randomly selected 50% of the segments and then used a test and validated the model's output on the remaining segments. The overall proposed scheme is demonstrated in Algorithm 1.

### 3.1. Statistical Tests for ARCH/GARCH Effect

GARCH models can only be used when the data are volatile. We need to verify the volatility of data before using any GARCH models. We use various tests to explore ECG segments' statistical properties to examine whether GARCH family models provide an efficient ECG signals modeling. One of the approaches is by measuring histograms for verifying data distribution. Kurtosis is the indicator of peaks in the data distribution, and skewness is a symmetrical representation of a mean distribution. The series is volatile when the kurtosis value is greater than 3 and is skewed to either the left or the right. In simple terms, the heavy-tailed distribution indicates that the probability of encountering large deviations from the mean is higher than in the case of normal distribution. Kurtosis and skewness measurements are used as follows:

(7) $$\begin{array}{c} \text{Kurtosis}=\frac{E{\left(x-\mu \right)}^{4}}{\sigma^{4}},\\ \text{Skewness}=\frac{E{\left(x-\mu \right)}^{3}}{\sigma^{3}}, \end{array}$$

where *μ* and *σ* are the mean and the standard deviation of *x*. Another method for testing ARCH/GARCH effects is the ARCH/GARCH test suggested by Engle [33]. This approach tests a null hypothesis that the ARCH/GARCH effect does not exist. Besides, this statistical test is asymptotically distributed as chi-square. The final test form is based on the Wilcoxon signed-rank test, which is a nonparametric statistical test to assess if two populations are similar without assuming that they obey the normal distribution. The null hypothesis of the test is that the output indicators are equivalent or comparable to populations for GARCH models versus ECG segments. The test statistics, *W*, is the total of the positive difference ranks (i.e., *x* − *y*) between the two samples. We set 0.05 as the level of significance for the test. If the “*P* value” is less than 0.05, we can conclude that the significance level of the null hypothesis is violated. This test is given as follows:

(8) $$\begin{array}{c} z\left(x,y\right)=\frac{\left(W-n\left(n+1\right)/4\right)}{\sqrt{\left(n\left(n+1\right)\left(2n+1\right)-\text{tieadj}\right)/24}}, \end{array}$$

where *n* corresponds to the sample size of the *x* − *y*. Signrank uses [tie_*r*_ank, tieadj]=tiedrank(abs(diffxy), 0,0, epsdiff) to get the tie adjustment value tieadj for the two-sample event.

The article "ECG Signal Modeling Using Volatility Properties: Its Application in Sleep Apnea Syndrome" was published in 2021. Journal: J Healthc Eng.

### 3.2. Order Selection

An ARIMA(*p*, *d*, *q*) model can be constructed by visually inspecting the autocorrelation function (ACF) and partial autocorrelation function (PACF). However, using objectively defined parameters such as Akaike information criteria (AIC) and Bayesian Information Criterion (BIC) is a more objective approach to determine *p*, *q*, and *d* of an ARIMA(*p*, *d*, *q*) method. These information criteria are statistical model fit measures [37]. They provided a set of results and assessed the relative fitness of the model of a number of previously developed mathematical models. Each of these criteria defines a *c*_*n*_(*k*) formula, where *k* denotes the number of model parameters and *n* the number of observations. The model with the fewest parameters, *k*, is called the best fit, and the quantity *c*_*n*_(*k*) is the smallest. The AIC [38] is an information processing method focused on the principle of entropy. The AIC's main concept is to look at the model's difficulty and its fit to the sample data and come up with a score that combines the two. Its formula is [37].

(9) $$\begin{array}{c} \text{AIC}:c_{n}\left(k\right)=2.\left(\frac{k}{n}\right)-2\;\ln\frac{\left(L\right)}{n}, \end{array}$$

where *L* denotes the likelihood function, *k* denotes the number of model parameters, and *n* denotes the number of observations.

Schwarz [39] provides the BIC:

(10) $$\begin{array}{c} \text{BIC}:c_{n}\left(k\right)=k.\ln\frac{\left(n\right)}{n}-2\ln\frac{\left(L\right)}{n}. \end{array}$$

Both of these criteria have advantages and disadvantages. Shibata [40] studied the asymptotic properties of the AIC estimation, concluding that the AIC estimate is inconsistent and asymptotically overestimates *k* with a nonzero probability. BIC is known to underestimate *k* [41]. Therefore, in the present study, we used the BIC criterion. The model with the lowest amount of BIC value is chosen as the most suitable match.

The article "ECG Signal Modeling Using Volatility Properties: Its Application in Sleep Apnea Syndrome" was published in 2021. Journal: J Healthc Eng.

### 3.3. Evaluation Methods of Model Sufficiency

There is usually no common criterion for evaluating a model's forecast output and comparing it with other benchmark models [42]. Since there are no common parameters for measuring errors, various error metrics were used to verify the proposed model's efficacy. The model performance evaluation is done in this analysis by comparing the expected values with their corresponding observed values using traditional performance metrics, such as mean square error (MSE), root mean square error (RMSE), mean absolute error (MAE), and mean absolute percentage error (MAPE) based on the following equations:

(11) $$\begin{array}{c} \text{MSE}=\frac{1}{N}\sum_{i=1}^{N}{\left(X_{i}-\hat{X_{i}}\right)}^{2}, \end{array}$$

(12) $$\begin{array}{c} \text{RMSE}=\sqrt{\frac{1}{N}\sum_{i=1}^{N}{\left(X_{i}-\hat{X_{i}}\right)}^{2}}, \end{array}$$

(13) $$\begin{array}{c} \text{MAE}=\frac{1}{N}\sum_{i=1}^{N}\left|X_{i}-\hat{X_{i}}\right|, \end{array}$$

(14) $$\begin{array}{c} \text{MAPE}=\frac{1}{N}\sum_{i=1}^{N}\left|\frac{X_{i}-\hat{X_{i}}}{X_{i}}\right|\times 100\%, \end{array}$$

where *N* is the number of samples in one segment and *X*_*i*_, $\hat{X_{i}}$ are observed and predicted values in one segment. These errors are advisable for predicting time series with the same scale and the same data processing procedures. The model with the smaller value of MSE, RMSE, MAE, and MAPE is selected as the best model. MAE and RMSE calculated the average of forecast errors over a sample size *n*. MAE and RMSE have the analyzed signal units. MAPE, which is a dimensionless quantity, assesses the predictive model's accuracy. In statistics, MAPE calculates the precision of the prediction of a forecasting system and is typically expressed as a percentage. The predictive potential of the proposed ARIMA-EGARCH model was assessed by using equations (11)–(14).

## 4. Numerical Results

### 4.1. Data

In this study, the Physionet Apnea-ECG dataset (https://www.physionet.org/physiobank/database/apnea-ecg/) was used [43, 44] because of its availability and widespread use in the literature. Recordings were obtained from 32 people (25 men and 7 women). A total of 35 recordings sampled at 100 Hz from normal subjects and subjects with OSA were used. All signals were segmented into one-minute segments, and each segment was labeled as apnea or normal by physicians. Recordings varied in length from slightly less than 7 hours to almost 10 hours and were divided into three groups:

  Apnea group: with 100 minutes or more of apnea, the mean age is 50 years. The range of age is 29–63 years.
  Borderline group: with 10–96 minutes of apnea, the mean age is 46 years. The range of age is 39–53 years.
  Healthy group: with 5 minutes or fewer of apnea, the mean age is 33 years. The range of age is 27–47 years.

The article "ECG Signal Modeling Using Volatility Properties: Its Application in Sleep Apnea Syndrome" was published in 2021. Journal: J Healthc Eng.

### 4.2. Results

The first step in the modeling method is to approximate the mean of the data. In the literature, numerous mean equation models have been studied. Among these latest processes, which have been suggested, the ARIMA-type model was one of the most commonly used approaches in the literature due to its simplicity of execution and its well-known ability to predict and forecast. Therefore, this article applies the ARIMA model as the mean equation. ECG signals are nonstationary. To implement the aforementioned time series models on ECG signals, we must ensure that the time series is stationary. If the data are nonstationary, then the first difference is used to transform it. Plotting the first difference data will show whether the data have been converted into a stationary sequence. The second difference is taken if it is still not stationary. Model fittings can be made once the time series is stationarity. In the ARIMA model, this mechanism determines the differentiating parameter “*d*.” As “*d*” is typically less than 2, we created the new time series by first and second differentiating the ECG signal. To find *p*, *q*, and *d* order, several combinations of ARIMA(*p*, *d*, *q*) are tested by the BIC, and the model with the smallest amount of BIC is selected. Results show that ARIMA(5, 2, 4) has the minimum amount of BIC for most segments. So, we consider ARIMA(5, 2, 4) for all segments.

Since the ECG signal is nonstationary, both the mean and percentiles of the data are different at varying periods. This means that the residual series differs over time, and the constant variance concept of the standard time series models is broken. This further proves that the volatility model is essential. The GARCH models can only be used on volatile data. That is why a histogram is plotted to analyze whether or not ECG segments follow a normal distribution.  Figure 1 shows the histogram for one ECG segment.

Then, kurtosis is determined. The minimum and the maximum kurtosis for all ECG segments are 5.1479 and 281.4540, respectively. It is evident from the minimum value that all measured kurtosis is higher than the value of three predicted for Gaussian distribution and histogram skewed to the right. Kurtosis values indicate that ECG segments have heavy tail characteristics and are not normally distributed. We also performed a Wilcoxon signed-rank test.  Table 1 gives the “*h,*” “*P* value”, and “Stat” for the test. “*h* = 1” indicates a rejection of the null hypothesis, and “*h* = 0” indicates a failure to reject the null hypothesis at the 5% significance level. “Stat” has information about the test statistic. The “*P* values” of the statistical test for the ECG segments versus GARCH are more than 0.05, as shown in Table 1. This indicates that the ECG segments are statistically similar to GARCH models. We also used the ARCH/GARCH test suggested with Engle. Results of Engle's test are shown in Table 2,

“H” is the Boolean decision variable. “1” suggests a null hypothesis rejection that there is no ARCH/GARCH effect. “Stat” displays ARCH/GARCH test statistics, and the “critical value” calculates the critical value of the chi-square distribution. If the “Stat” is below the “critical value” point, at a meaning level equal to 5%, there is no GARCH effect. However, if “Stat” is more than “critical value,” it formally shows clear evidence for GARCH in this time sequence. We applied the ARCH/GARCH test to all of the ECG signals in the databases. Because of the limited space, we demonstrate in this section the results of some representative signals. We should also remember that the simulated results are identical for different ECG signals. As shown in Table 2, for all signals, “H” is 1, and “Stat” is more than “critical value,” which means the null hypothesis is rejected, and therefore, the ECG signals have an ARCH/GARCH effect. Finally, visual validation is also performed between the histogram of ECG signals and the GARCH family models.  Figure 2 shows ECG segment histograms and Gaussian distribution function with the estimated mean and standard deviation from the data and a corresponding GARCH model histogram.

The article "ECG Signal Modeling Using Volatility Properties: Its Application in Sleep Apnea Syndrome" was published in 2021. Journal: J Healthc Eng.

From Figure 2, it is evident that there is high accuracy between the histogram of ECG segments and the GARCH model. Compared to Gaussian, the studied distribution is sharper and has a zero peak with a heavier tail. We also plot the cumulative distribution function (CDF) of ECG segments and the corresponding GARCH model in Figure 3.

It is evident from Figure 3 that ECG segments and the GARCH data are from the same CDF. Considering the results in Tables 1 and 2 and Figures 1–3, we find an ARCH/GARCH effect in all examined ECG segments. It should be again reported that the results of modeling various ECG signals are identical. However, only a few results are shown here. Hence, we proposed GARCH family models and demonstrated that they were a suitable representation of ECG segments.

The literature is comprehensive on the GARCH family models. However, we limit our study to the three more common models for compactness, namely, GARCH, EGARCH, and GJR-GARCH. Estimating the volatility model requires order selection and parameter estimation, similar to the ARIMA model. Again, to find the proper order of GARCH, EGARCH, and GJR-GARCH models, several combinations were tested by the BIC, and the models with the smallest amount of BIC were selected.

The article "ECG Signal Modeling Using Volatility Properties: Its Application in Sleep Apnea Syndrome" was published in 2021. Journal: J Healthc Eng.

Results show that GARCH(1,4), GJR-GARCH(1,5), and EGARCH(1,5) have the minimum BIC for most segments. So, we consider GARCH(1,4), GJR-GARCH(1,5), and EGARCH(1,5) for all segments. We calculated the log-likelihood amount of GARCH, GJR-GARCH, and EGARCH to find the best model among the others. We also computed log-likelihood for ARIMA-GARCH, ARIMA-GJR-GARCH, and ARIMA-EGARCH. The model with the maximum amount of log-likelihood was selected as a proper model. The results are illustrated in Figure 4. As is evident from Figure 4, GJR-GARCH and ARIMA-EGARCH have a maximum amount of log-likelihood. Finally, in each segment, the maximum likelihood estimation (MLE) was used to identify model coefficients. MLE is applied to both ARIMA and GARCH models.

In the next step, we validated our proposed method on the remaining ECG segments, which were not used in the model estimation step. We run ARIMA and GJR-GARCH models on the Physionet Apnea-ECG database and compared the ARIMA-EGARCH model results with these models using MSE, RMSE, MAE, and MAPE. The reason for choosing these models is that linear models such as AR, MA, and ARMA are coarse estimations of real-world systems and usually have poor performance in forecasting the evolution of nonstationary and nonlinear processes; ARIMA model is usually used to model these patterns [31]. So, we considered the ARIMA model as the first model for comparison. On the other hand, we showed that ECG signals were heteroskedastic; GARCH family models can be used to model them. Since the log-likelihood of GJR-GARCH had maximum value, we selected GJR-GARCH as the second model. Average and standard deviation of MSE, RMSE, MAE, and MAPE based on the assessment criteria 11, 12, 13, and 14 for ARIMA, GJR-GARCH, and ARIMA-EGARCH models on apneic and normal ECG segments are presented in Tables 3 and 4, respectively.

Tables 3 and 4 demonstrate that in terms of averaged MSE, RMSE, MAE, and MAPE, the proposed ARIMA-EGARCH model outperforms all other models in modeling both apnea and normal ECG signals. The lowest prediction error value reflects the superiority of the proposed ARIMA-EGARCH model over the ARIMA model and the GJR-GARCH model.

The graphical validation of our model on the sample test data is illustrated in Figures 5 and 6 for sample apneic and normal ECG segments using three different models, respectively. For better understanding, we only show the 500 first samples of each segment in figures.

The article "ECG Signal Modeling Using Volatility Properties: Its Application in Sleep Apnea Syndrome" was published in 2021. Journal: J Healthc Eng.

Figures 5 and 6 show that the ARIMA-EGARCH model can best model both sudden and slow transients in apneic and normal ECG signals. Moreover, if we only consider slow changes in the ECG signal, we can see that a linear approach such as ARIMA cannot predict slow changes, but a nonlinear method like GJR-GARCH can predict almost slow changes (white noise). These findings confirm our claim that EGARCH models improve the estimation made by ARIMA and a combination of ARIMA and EGARCH models can complete each other in ECG signal modeling.

### 4.3. Comparison with Other Models

In this section, the performance of the selected model is compared with other models proposed in the literature. Since the results obtained from the same sample must be compared for meaningful comparison, we must compare our results with the results of models that used the Physionet Apnea-ECG. As mentioned in the Introduction, only a few researchers used models to detect apnea [26–28], and these articles fit models to QRS complexes and not the entire ECG. Therefore, we can not compare our results with them. On the other hand, these articles used the model's parameters to detect sleep apnea, and they did not compare the estimated results with the actual ECG signal. Only Hu et al. [30] proposed a mathematical model for apneic and normal ECG signals. Therefore, to show our model's capability, we compared our results with this article. Tables 5 and 6 compare RMSEs and MAEs from ARIMA-EGARCH with ARCH(1) [30], GARCH(1,1) [30], Student-t GARCH(1,1) [30], Integrated GARCH(1,1) [30], and Student-t Integrated GARCH(1,1) [30] for apneic and normal segments, respectively.

## 5. Discussion and Conclusion

This article describes a method for mathematical modeling of the ECG signal. Although the forecasting of time series is a vast research area, it can be classified into short- and long-term predictions. Short-term forecasting can also be split into mathematical modeling and physiological modeling. The mathematical-based forecasting model uses mathematical representation and dynamic variations to predict the future status of the time series of the process that underlies it. It should be clear that no apnea detection method is provided in this article. We have shown that ECG signals are heteroskedastic, which means the conditional variance is not constant. In the literature, ECG volatility and heteroskedasticity during apnea are underestimated. Thus, we used this characteristic to model ECG signals.

The proposed ARIMA-EGARCH can model the mean and volatility of ECG signals in sleep apnea syndrome. This model can cover both linear and nonlinear characteristics of ECG signals. Using BIC, the best orders of the ARIMA and EGARCH models were estimated. The model parameters were approximated using the maximum likelihood estimation method. Finally, some metrics, including MSE, RMSE, MAE, and MAPE, between the actual and estimated ECG signals were calculated. The method is validated and compared to other methods, using recordings from the Physionet Apnea-ECG database containing ECG segments during sleep apnea and normal breathing. Visual quality and objective quality of the proposed approach were achieved in terms of MSE, RMSE, MAE, and MAPE. Since the results obtained from the same sample must be compared for meaningful comparison, we must compare our results with the results of models that used the Physionet Apnea-ECG. So, we compared our proposed model with models in [30] (see Tables 4 and 5). As it can be inferred from Tables 4 and 5, the proposed ARIMA-EGARCH model outperforms the other existing models for sleep apnea modeling. Experimental findings show that the ARIMA-EGARCH model can estimate both normal and apneic ECG signals. Our results are robust for selecting performance assessment criteria.

The article "ECG Signal Modeling Using Volatility Properties: Its Application in Sleep Apnea Syndrome" was published in 2021. Journal: J Healthc Eng.

The proposed model has some advantages. The estimated model's parameters can be used as features for the automatic detection of sleep apnea [45]. Moreover, one of the current widespread therapies in sleep apnea is continuous positive airway pressure (CPAP) that blows constant air at a fixed pressure. ECG model can be used in CPAP machines in order to blow air only when apnea occurs.

## Figures and Tables

**Figure 1:** Histogram for an ECG segment.

**Figure 2:** Histograms of ECG segment, corresponding GARCH model, and Gaussian distribution of (a) an apneic segment and (b) a normal segment.

**Figure 3:** Comparison of cumulative distribution function (CDF) of ECG segments (solid line) and CDF of GARCH data (dash line) for (a) apneic and (b) normal segments.

**Figure 4:** The likelihood values of (a) GARCH, EGARCH, and GJR-GARCH models; (b) ARIMA-GARCH, ARIMA-EGARCH, and ARIMA-GJR-GARCH models.

**Figure 5:** Fitting results using ARIMA, GJR-GARCH, and ARIMA-EGARCH models on a sample apneic ECG segment (blue line: ECG data; redline: estimated data).

**Figure 6:** Fitting results using ARIMA, GJR-GARCH, and ARIMA-EGARCH models on normal ECG data (blue line: ECG data; redline: estimated data).

**Algorithm 1:** The proposed procedure for modeling apneic and normal ECG signals.

**Table 1:** Results of the Wilcoxon signed-rank test.

Signal	*H*	Stat	*P* value
Signal 1	0	38	0.3223
Signal 2	0	41	0.1934
Signal 3	0	45	0.0840
Signal 4	0	38	0.3223
Signal 5	0	45	0.0840
Signal 6	0	37	0.3750
Signal 7	0	41	0.1934
Signal 8	0	41	0.1855

The article "ECG Signal Modeling Using Volatility Properties: Its Application in Sleep Apnea Syndrome" was published in 2021. Journal: J Healthc Eng.

**Table 2:** Results of Engle's test for the existence of ARCH/GARCH effects.

Signal	*H*	Stat	Critical value
Signal 1	1	2.6848*e* + 3	3.8415
Signal 2	1	3.1229*e* + 3	3.8415
Signal 3	1	3.1219*e* + 3	3.8415
Signal 4	1	3.2108*e* + 3	3.8415
Signal 5	1	3.1211*e* + 3	3.8415
Signal 6	1	2.8983*e* + 3	3.8415
Signal 7	1	3.2584*e* + 3	3.8415
Signal 8	1	3.2659*e* + 3	3.8415

**Table 3:** Comparison of MSEs, RMSEs, MAEs, and MAPEs from different models estimated for apnea segments.

	ARIMA		GJR-GARCH		ARIMA-EGARCH	
	Ave	Std	Ave	Std	Ave	Std
MSE	0.0181	0.0133	0.2032	0.7924	**0.0177**	0.0129
RMSE	0.1232	0.0543	0.2990	0.3378	**0.1216**	0.0535
MAE	0.0666	0.0282	0.0736	0.0140	**0.0613**	0.0255
MAPE	13.6081%	42.5486%	42.3760%	678.0458%	**4.0841%**	15.9423%

Ave = average, Std = standard deviation.

**Table 4:** Comparison of MSEs, RMSEs, MAEs, and MAPEs from different models estimated for normal segments.

	ARIMA		GJR-GARCH		ARIMA-EGARCH	
	Ave	Std	Ave	Std	Ave	Std
MSE	0.0235	0.0131	0.6792	4.0802	**0.0230**	0.0128
RMSE	0.1454	0.0490	0.4477	0.6928	**0.1437**	0.0484
MAE	0.0810	0.0250	0.0962	0.0526	**0.0754**	0.0226
MAPE	16.1331%	97.8801%	18.5205%	161.6340%	**4.7286%**	29.5338%

Ave = average, Std = standard deviation.

**Table 5:** Comparison of RMSEs and MAEs from ARIMA-EGARCH with other existing models for apnea segments.

Method	RMSE	MAE
ARCH(1) [30]	0.6614	0.5876
GARCH(1,1) [30]	0.6636	0.5808
Integrated GARCH(1,1) [30]	0.6325	0.5725
Student-t GARCH(1,1) [30]	0.6497	0.5625
Student-t Integrated GARCH(1,1) [30]	0.6551	0.5638
ARIMA(5,2,4)-EGARCH(1,5)	**0.1216**	**0.0613**

**Table 6:** Comparison of RMSEs and MAEs from ARIMA-EGARCH with other existing models for normal segments.

Method	RMSE	MAE
ARCH(1) [30]	0.6482	0.5652
GARCH(1,1) [30]	0.6508	0.5618
Integrated GARCH(1,1) [30]	0.7133	0.5843
Student-t GARCH(1,1) [30]	0.7347	0.5785
Student-t Integrated GARCH(1,1) [30]	0.7212	0.5841
ARIMA(5,2,4)-EGARCH(1,5)	**0.1437**	**0.0754**

## Data Availability

In this study, the Physionet Apnea-ECG dataset is available at https://www.physionet.org/physiobank/database/apnea-ecg/ was used.
